# Efficient Johnson-S_B_ Mixture Model for Segmentation of CT Liver Image

**DOI:** 10.1155/2022/5654424

**Published:** 2022-04-14

**Authors:** Yueqin Dun, Yu Kong

**Affiliations:** ^1^School of Electrical Engineering, University of Jinan, Jinan, Shandong, China; ^2^Department of Medical Imaging, Shandong Medical College, Jinan, Shandong, China

## Abstract

To overcome the problem that the traditional Gaussian mixture model (GMM) cannot well describe the skewness distribution of the gray-level histogram of a liver CT slice, we propose a novel segmentation method for liver CT images by introducing the Johnson-SB mixture model (J_SB_MM). The Johnson-SB model not only has a flexible asymmetrical distribution but also covers a variety of other distributions as well. In this article, the parameter optimization formulas for J_SB_MM were derived by employing the expectation-maximization (EM) algorithm and maximum likelihood. The implementation process of the J_SB_MM-based segmentation algorithm is provided in detail. To make better use of the skewness of Johnson-SB and improve the segmentation accuracy, we devise an idea to divide the histogram into two parts and calculate the segmentation threshold for each part, respectively, which is called J_SB_MM-TDH. By analyzing and comparing the segmentation thresholds with different cluster numbers, it is illustrated that the segmentation threshold of J_SB_MM-TDH will tend to be stable with the increasing of cluster number, while that of GMM is sensitive to different cluster numbers. The proposed J_SB_MM-TDH is applied to segment four randomly obtained abdominal CT image sequences, and the segmentation results and robustness have been compared between J_SB_MM-TDH and GMM. It is verified that J_SB_MM-TDH has preferable segmentation results and better robustness than GMM for the segmentation of liver CT images.

## 1. Introduction

Liver cancer is a common malignant neoplasm worldwide, and the incidence of primary liver cancer is still on the rise at the global level [1]. The accurate understanding of the shape of the liver, the location and size of lesions in the liver tissue, and the relationship between the liver and surrounding blood vessels can help doctors to develop more effective treatment options. In addition, accurate liver segmentation is also conducive to three-dimensional reconstruction for liver and virtual surgery. At present, manual delineation of each slice by experts is still the standard clinical practice for liver demarcation [2]. Because the segmentation of organs and lesions has to be carried out layer by layer in CT slices, it is pretty cumbersome and time-consuming for doctors or experts to do this repetitive work.

In practice, CT slices are grayscale images. The pixels in the image reflect the X-ray absorption coefficient of the corresponding voxels. Black areas represent low absorption areas, that is, low-density tissues and organs of human body, such as lungs; white areas represent high-absorption areas, that is, high-density body parts, such as bones. The absorption value in CT images is given in Hounsfield units (HUs). Compared with ordinary X-ray images, CT images have a higher density resolution. Therefore, CT images can better show organs composed of soft tissue, such as lung, liver, gallbladder, pancreas, and pelvis, and can well demonstrate pathological changes in the tomography image. At present, the original pixel size of the abdominal CT image is 512 × 512, and the HU value of the liver varies widely. For example, a healthy liver has smooth contours and uniform density, and the absorption values are 60 ± 6 HU (or 64 ± 5 HU). However, when the liver has about 80% steatosis, the absorption values will be reduced to about −50 HU. In contrast, the density of the liver parenchyma will increase due to the accumulation of iron in patients with hemochromatosis, whose CT scan showed that the liver parenchyma was clearly dense and bright, with an absorption value as high as +140 HU (so-called white liver) [3]. There is no doubt that it is quite difficult to accurately segment the liver within such a large gray range.

To solve the above problems, many scholars have proposed a variety of liver CT image segmentation methods [4–7]. Some of these algorithms require human-computer interaction, such as active contour [8] and Livewire (intelligent scissors) [9, 10]. Some are semi-automatic, for example, graph-cut [11] and region growth [12, 13] methods. Some other methods focusing on fully automatic segmentation include statistical shape models (SSMs) [14, 15] and thresholding algorithm [16]. Neural network algorithms aiming to achieve automatic feature extraction have also been applied to the segmentation of medical images in recent years [17, 18]. The ultimate common goal of different methods is to segment images accurately and automatically, but this goal is still a bottleneck problem in liver CT image segmentation, due to the complexity of abdominal CT images and the differences between different liver morphologies. In this study, we aim to study on the finite mixture model (FMM), one kind of threshold segmentation algorithm, to improve the segmentation accuracy of liver CT images, and try hard to segment automatically at the same time.

According to the idea of the threshold segmentation algorithm, if the grayscale threshold of the liver in the CT slice can be accurately determined, it is possible to realize the liver segmentation automatically. In 1893, Karl Pearson made an experiment using the method of moments to fit a mixture of two normal components to the crabs' data, which proved the FMM could improve the accuracy of clustering [19]. Since then, FMM was adopted to improve the accuracy of threshold segmentation methods. In 1972, Chow and Kaneko applied FMM in medical images to segment the left ventricle from cine angiograms with two Gaussian distributions [20].

There are two core points in FMM, one is the selection of the probability density function of the mixed components and the other is the parameter estimation of the mixture model. The most common mixed component probability distribution used in FMM is the Gaussian distribution, because in many cases there is a normal distribution in univariate and multivariate data. Therefore, the Gaussian mixture model (GMM) has been widely used in the segmentation of the images [21–24]. In addition to the Gaussian distribution, gamma distribution, Student's t distribution, exponential distribution, and Rayleigh distribution also commonly appear in FMM [25–27], and their probability density diagrams with different parameters are shown in Figure 1, respectively.

The upper, middle, and lower slices of the liver CT image sequence are shown in Figures 2(a)∼2(c)), respectively. Figures 2(d)∼2(f) give the corresponding gray-level histograms of Figures 2(a)∼2(c)). Although the peak shape of gray-level histogram has symmetry to some extent, its asymmetry is also very obvious, which is different from the symmetric characteristic of Gaussian distribution and the asymmetric characteristic of the exponential, Rayleigh distribution, etc. Therefore, it is very difficult to fit the peak shape accurately with any single distribution shown in Figure 1.

To solve the problem, many researchers have focused on forming a mixture model using distribution functions that can better fit the shape of a single peak. The research ideas mainly concentrate on the following three kinds of mixture models.

The first kind of mixture model is forming an asymmetric generalized Gaussian distribution (AGGD) by introducing shape parameters or functions into the generalized normal distribution to describe the skew characteristic [28, 29], so that it can describe not only a symmetric distribution but also an asymmetric distribution. However, the expression of the AGGD is complicated by embedding the gamma function. In the case of using the EM algorithm for maximum-likelihood estimation (MLE), all AGGD parameters in the mixture model are represented by highly nonlinear equations, which makes the numerical solutions cumbersome and sensitive to initial EM values [30].

Combining Gauss with other distributions to form a new model is the second idea. Wilson selected two Gaussian distributions and one uniform distribution to fit the low-gray and high-gray regions of the brain MRA data histogram, respectively [31]. Hassouna proposed a linear combination of a finite mixture model using one Rayleigh distribution and two Gaussian distributions [32]. Hence, for different problems, people need to determine in advance which existing models can be used to form a new probability distribution model, and the number of each distribution also needs to be determined in advance. Therefore, this kind of model is not flexible, and it is also difficult to realize segmentation automatically.

The third way is to combine the components of the mixed model with the non-Gaussian distribution. Lee and McLachlan introduced a finite mixture of canonical fundamental deviation *t* (CFUST) distributions for asymmetric and possibly long-tailed clusters [33]. Sefidpour and Bouguila proposed and investigated the segmentation of spatial color images using the Dirichlet and Beta-Liouville distributions [34]. The normal inverse Gaussian distribution (NIG) is chosen by Karlis and Santourian to deal with skewed subpopulations [35]. Franczak et al. studied the asymmetric Laplace distribution (ALD) for clustering and classification [36]. NIG and ALD belong to the family of generalized hyperbolic (GH) distributions designed by Barndorff-Nielsen [37]. Browne and McNicholas extended a special case for the generalized hyperbolic distribution [38]. Wraith and Forbes studied the properties of these distributions in multiscale and their application in multivariate clustering [39]. Although there are many combination methods of non-Gaussian distribution, only a few methods are used for the segmentation in medical images, especially in liver CT images. Therefore, the study on the segmentation of liver CT images still needs further research.

Considering the asymmetric skew characteristic of the gray histogram of the liver CT image, and inspired by the skew characteristic of Johnson-S_B_ distribution, we propose a novel mixture model with the combination of Johnson-S_B_ distribution to segment the liver CT image. In the following paper, the Johnson-S_B_ mixture model and the optimized parameters with the EM algorithm are introduced firstly in Section 2. Secondly, Section 3 gives the implementation details of the segmentation algorithm based on the Johnson-S_B_ mixture model, and the effects of cluster number on the segmentation threshold are also analyzed and compared between GMM and Johnson-S_B_ mixture model in this section. Then, the segmentation experimental results of four randomly obtained abdominal CT image sequences from different image databases are provided in Section 4. Finally, conclusions are drawn in Section 5.

## 2. Finite Johnson-S_B_ Mixture Model

In 1949, Johnson deduced a curve system called the Johnson system, which contains Johnson-S_B_, Johnson-S_L_, and Johnson-S_U_. The symbol *S*_L_ means “log-normal system,” *S*_B_ means “bounded system,” and *S*_U_ means “unbounded system” [40]. The Johnson system can closely approximate many continuous distributions by one of the three functional forms, so it is very flexible to fit variety curves. Many of the commonly used continuous distributions, such as normal, log-normal, gamma, beta, and exponential, are special cases of the Johnson system; therefore, it has more advantages to fit curves with the Johnson system than any other single distribution [41].

### 2.1. Johnson-S_B_ Distribution

Johnson-S_B_ is one of the three distributions of the Johnson system. It corresponds to the distribution of a continuous random variable *x* in which a particular transformation is applied to obtain a normal distribution. The transformation is as follows:

(1) $$\begin{array}{c} z=\gamma +\delta \text{ln}\left(\frac{x-\xi }{\lambda +\xi -x}\right), \end{array}$$

where *x* is a given continuous random variable. In this study, *x* is the grayscale value of the pixel in the CT image. *x* ∈ (*ξ*, *ξ* + *λ*), *ξ* = min (*x*), *λ* = max (*x*) − min (*x*), and *γ* and *δ* are shape parameters, *δ* *>* 0, *γ* ∈ (−∞, +∞). *Z* is a standard normal random variable, and its probability density function is as follows:

(2) $$\begin{array}{c} \text{p}\left(z\right)=\frac{1}{\sqrt{2\pi }}.e^{-\;z^{2}/2}. \end{array}$$

We write

(3) $$\begin{array}{c} \text{z}=\gamma +\delta f\left(y\right),\;y=\frac{x-\xi }{\lambda +\xi -x}\text{,}\;\text{and}\;f\left(y\right)=\text{ln}\left(\frac{x-\xi }{\lambda +\xi -x}\right), \end{array}$$

where *z* is the inverse function of *y*.

According to the transformations of continuous random variable,

(4) $$\begin{array}{c} p\left(y\right)=\delta f^{\prime }\left(y\right)p\left(z\right)=\frac{\delta }{\sqrt{2\pi }}.f^{\prime }\left(y\right).e^{-\;1/2{\left[\gamma +\delta f\left(y\right)\right]}^{2}}. \end{array}$$

Then, the probability density function (PDF) with regard to  *x* is as follows:

(5) $$\begin{array}{c} \text{p}\left(x\right)=\left\{\frac{\delta }{\sqrt{2\pi }}.\frac{\lambda }{\left(x-\xi \right)\left(\lambda +\xi -x\right)}.e^{-\;1/2{\left[\gamma +\delta \text{ln}\left(x-\xi /\lambda +\xi -x\right)\right]}^{2}}.\right. \end{array}$$

Figure 3 shows some typical probability density function curves of Johnson-S_B_ with different parameters. The range of horizontal coordinates is from 0 to 255, and the vertical coordinates are the corresponding probability density function values. Figure 3(a) presents the curves with different *δ* and *γ* = 0, and it is a normal distribution in the middle. Figures 3(b)∼3(e) present the curves with different *δ* and *γ* = 0, respectively, and they have better skew characteristics, especially at the two ends of the abscissa. It can be seen that *γ* controls the position of the function, and the distributions of the function are normal distribution, negatively skewed distribution, and positively skewed distribution when *γ* = 0, *γ* *>* 0, and *γ* *<* 0, respectively.

### 2.2. Johnson-S_B_ Mixture Model (J_SB_MM) and Optimizing Parameters

#### 2.2.1. Johnson-S_B_ Mixture Model (J_SB_MM)

The finite mixture model (FMM) refers to the linear superposition of distribution functions of the same type but with different parameters. In the discrete case, the probability density function of a finite mixture distribution can be expressed as a p-dimensional random vector *X* [42].

(6) $$\begin{array}{c} \text{p}\left(x|\Theta \right)=\overset{K}{\underset{k=1}{\sum }}\Phi_{k}p_{k}\left(x|\theta_{k}\right), \end{array}$$

where *x* ⊂ X is the pixel grayscale value in the CT image, *θ*_*k*_ = (*δ*_*k*_, *γ*_*k*_), *p*_*k*_ (*x*|*θ*_*k*_) is the density of the *k*th component, and Θ = (Φ_1_,…, Φ_*k*_; *θ*_1_,…, *θ*_*k*_) is the vector of parameters. Note that *p* (*x| ***Θ**) in Eqn (3) defines a density that is called a *K*-component finite mixture density. Here, the weight of the *k*th mixing proportion Φ_*k*_ satisfies the following relations:

(7) $$\begin{array}{c} 0\leq \Phi_{k}\leq 1\;k=1,2,3,\ldots ,K, \end{array}$$

and

(8) $$\begin{array}{c} \overset{K}{\underset{k=1}{\sum }}\Phi_{k}=1. \end{array}$$

According to Eqn (3), the probability density of a Johnson-S_B_ mixture model is defined as follows:

(9) $$\begin{array}{c} \text{p}\left(x|\Theta \right)=\overset{K}{\underset{k=1}{\sum }}\Phi_{k}p_{k}\left(x|\delta_{k}\;,\gamma_{k}\right). \end{array}$$

Here,

(10) $$\begin{array}{c} p_{k}\left(x|\delta_{k}\;,\gamma_{k}\right)=\frac{\delta_{k}}{\sqrt{2\pi }}.\frac{\lambda }{\left(x-\xi \right)\left(\lambda +\xi -x\right)}.e^{-\;1/2{\left[\gamma +\delta \text{ln}\left(x-\xi /\lambda +\xi -x\right)\right]}^{2}}, \end{array}$$

is the probability density of a random variable *X* for a Johnson-S_B_ distribution with the parameters *δ*_*k*_  and *γ*_*k*_.

#### 2.2.2. Optimizing Parameters with EM Algorithm

The vector of parameters Θ typically introduced by the log-likelihood function is defined as follows:

(11) $$\begin{array}{c} L\left(\Theta \right)=\text{ln}p\left(X|\Theta \right)=\overset{N}{\underset{i=1}{\sum }}\text{ln}p\left(x_{i}|\Theta \right)=\overset{N}{\underset{i=1}{\sum }}\text{ln}\overset{K}{\underset{k=1}{\sum }}\Phi_{k}p_{k}\left(x_{i}|\delta_{k}\;,\gamma_{k}\right),=\overset{N}{\underset{i=1}{\sum }}\text{ln}\overset{K}{\underset{k=1}{\sum }}\Phi_{k}\frac{\delta_{k}}{\sqrt{2\pi }}.\frac{\lambda }{\left(x_{i}-\xi \right)\left(\lambda +\xi -x_{i}\right)}.e^{-\;1/2{\left[\gamma +\delta \text{ln}\left(x-\xi /\lambda +\xi -x\right)\right]}^{2}}. \end{array}$$

Here, *x*_*i*_ is the *i*th discrete grayscale value and *N* is the number of discrete dots of CT image.

The detailed derivation of the parameters given in equations (6)–(8) is presented in Appendix A.

## 3. Segmentation Algorithm Based on J_SB_MM

### 3.1. Implementation Details

There are mainly four steps to implement the segmentation algorithm based on J_SB_MM, and the details of each step in Algorithm 2 are introduced as follows.

#### 3.1.1. Obtaining the Approximate Gray Value (LV_A)

The Hounsfield unit (HU) value of liver tissue varies from patient to patient. In addition, the X-ray tube of the CT machine will age with longtime use, which results in the intensity decrease in the X-ray source. Therefore, the liver HU values of different CT image sequences are usually different. Clearly, it is not possible to identify all liver scan sequences with the same HU range value.

We can make full use of the continuity of CT scan section images to solve this problem. CT scans require patients to hold their breath during data collection, and this process usually takes no more than 20 seconds [43]. Therefore, in the same CT image sequence, the range of gray values between all liver slices varied a little. It is feasible to obtain the liver HU value of this sequence using the slice image with the largest liver area.

Figure 4(a) shows the frontal outline of the liver, and Figures 4(b)∼4(d) give the upper, middle, and lower slice images of the liver CT scan sequence, respectively. It can be seen that the liver is almost completely surrounded by the ribs, and the liver image at about 1/3 of the entire sequence is the largest one [44]. For example, if a complete sequence of CT scans of the liver has 90 slices, the liver slice near the 30th slice will be more significant than others.

Figures 5(a) and 5(c) show two liver slices taken from two different CT scan sequences, which locate at 1/3 of each sequence. Grayscale-level statistics were performed at about 1/4 of the body section, shown as the dotted line in Figures 5(a) and 5(c). The approximate grayscale value of the liver (LV_A) can be easily calculated after removing the grayscale values of black and white zones. Figures 5(b) and 5(d) are the corresponding gray-level histograms with a sampling width of 10 pixels for the positions shown as the dotted lines in Figures 5(a) and 5(c), respectively. Here, the horizontal coordinates are the grayscale values, and the vertical coordinates are the statistical numbers of the corresponding grayscale values. The grayscale values with maximum statistical numbers are 131 and 178 as shown in Figures 5(b) and 5(d), respectively, which are taken as the approximate grayscale value of the liver (LV_A) in Figures 5(a) and 5(c), respectively. It should be noted that the maximum statistical number of the grayscale value 0 should be omitted, although it is more than 2000, because it means the black zone and is useless for the segmentation of the liver.

#### 3.1.2. Finding the Maximum Gray Value (LV_M)

Although liver HU values do not change significantly during the scan process, there also exist some slight changes. To segment each slice accurately, it is necessary to further locate the maximum grayscale value of the liver (LV_M) close to the LV_A on the gray-level histogram of each slice.

For instance, Figure 6(a) shows the slice of the upper part of the liver CT sequence shown in Figure 5(c).  Figure 6(c) displays the slice of the lower part in the same sequence.  Figure 6(b) gives the gray-level histogram of Figure 6(a), and the gray-level histogram of Figure 6(c) is shown in Figure 6(d). Because the value of LV_A shown in Figure 5(d) is 178, the corresponding LV_M values of Figures 6(a) and 6(c) are 179 and 176, as shown in Figures 6(b) and 6(d), respectively. Here, it needs to be stated that we should choose the peak value closest to 178 as LV_M, because 178 is determined in Figure 5(d).

#### 3.1.3. Determining the Segmentation Points

The position of peak and skewness characteristics of the gray-level histogram of liver slices are uncertain and nonuniqueness, so it is difficult to take full advantage of the J_SB_MM in describing skewness if J_SB_MM is applied directly to fit the whole gray-level histogram. To make full use of the advantages of Johnson-S_B_ in describing the skew characteristics, we divided the gray-level histogram into the left and right parts at LV_M to ensure that the gray level of the liver is just at the boundary of the histogram, to improve the Johnson-S_B_ segmentation accuracy.

The LV_M of Figure 6(c) is 176. At the LV_M point, the gray-level histogram shown in Figure 6(d) is divided into the left part and the right part, and the grayscale values of the segmentation points are obtained using J_SB_MM to fit the gray-level histograms. Figures 7(a) and 7(b) give the fitting results of the left part and the right part, respectively. The grayscale value of the segmentation point of the left part is 157, which is the intersection of the two rightmost fitting curves shown in Figure 7(a). The grayscale value of the segmentation point of the right part is 190, which is the intersection of the two leftmost fitting curves shown in Figure 7(b). However, if there is a peak of one fitting curve appearing between the intersection point of the other two fitting curves and the LV_M, the grayscale value of this peak will be taken as the segmentation point, which can get better segmentation results. For example, the grayscale value of the segmentation point of the right part should be 188, because the grayscale value of the peak is 188, which appears before the intersection of 190. Therefore, the range of the grayscale value for liver segmentation in Figure 6(c) is set from 157 to 188, which is the range of the segmentation thresholds for Figure 6(c).

#### 3.1.4. Binarizing the Images and Processing with Mathematical Morphology

Mathematical morphology is a tool for extracting image components. Erosion, dilation, and filling are three basic morphological set transformations. These transformations involve the interaction between image and structuring element [45]. Figure 7(c) is obtained by binarizing Figure 6(c). The final boundary of the liver segmentation can be drawn as shown in Figure 7(d) after the procession of filling, erosion, and expansion algorithms in mathematical morphology.

### 3.2. Effect of Cluster Number on the Segmentation Thresholds

A key point of FMM is how to select the cluster numbers to realize a better fitting, and underfitting or overfitting may occur if the cluster number is selected inappropriately [46]. In this study, the cluster number means the number of curves in a cluster used to fit the gray-level histogram. To analyze the effect of different cluster numbers on segmentation thresholds, we choose two different slices to be segmented by GMM and J_SB_MM in the following Section 3.2.1 and Section 3.2.2, respectively. The initial location of the grayscale value is another consideration to affect the segmentation threshold. In this study, the initial locations are evenly arranged within the range of the grayscale values of the entire image.

#### 3.2.1. Segmentation Thresholds of GMM with Different Cluster Numbers

Table 1 gives the segmentation thresholds of the upper, middle, and lower slices from two different CT image sequences. By analyzing the segmentation thresholds with different cluster numbers *n*, it can be found that the segmentation thresholds are changeable with the change in *n*, while they do not tend to be stable with the increasing *n*. In this study, *n* denotes the cluster numbers used to fit the gray-level histogram, and *n* is the same as K in Algorithm 1.

To illustrate the effect on the segmentation results with different cluster numbers, we give some segmentation results of the upper slices of the sequences S1 and S2. Here, Figure 8 shows the threshold segmentation results of the upper slices with *n* = 6, 8, 10, 12, and 14 using GMM, respectively. The first row and the second row give the segmentation results and thresholds for the upper slice of the first sequence S1. The third row and the fourth row give the results and thresholds for the upper slice of the second sequence S2.

By comparing the segmentation results in the first row, it is not difficult to find that the results of the first three columns with *n* = 6, 8, and 10 are similar, because the three segmentation results include some other organs that do not belong to the liver. Although the segmentation result in the fourth column with *n* = 12 only includes the liver, the segmentation result is a little smaller liver than that of the fifth column with *n* = 14. Therefore, the segmentation result with *n* = 14 is relatively more reasonable by comparing with the other four results for the first sequence.

Comparing the results of row 3 for the second sequence, it is obvious that the results of the first two columns with *n* = 6 and 8 are not correct, and the segmentation result of the third column with *n* = 10 is a little smoother than that of the fourth one with *n* = 12, while the segmentation result of the fifth column with *n* = 14 turns to be rougher boundary due to overfitting. Thus, the better segmentation result can be obtained when *n* is 10 for the second sequence. As can be seen from Figure 8, the segmentation results of GMM are sensitive to cluster numbers, and it is not easy for GMM to use fixed cluster number to get accurate segmentation results, which is a difficulty in the application of GMM, especially for a large number of images that need to be segmented.

Here, it is needed to be stated that the red contours in the figures in Figure 8 indicate the error zones of the segmentation. It is the same meaning in the following figures.

#### 3.2.2. Segmentation Thresholds of J_SB_MM with Different Cluster Numbers

Figures 9∼11 give the segmentation thresholds and the results of the upper, middle, and lower slices of the first liver CT sequence S1, and here, the segmentation thresholds are obtained with J_SB_MM-TDH, which means the gray-level histogram is divided into left and right parts, and it is denoted as thresholds of dividing histogram (TDH). While thresholds of whole histogram (TWH) mean that the segmentation thresholds are obtained with J_SB_MM under the whole gray-level histogram, and it is denoted as J_SB_MM-TWH. The segmentation results of J_SB_MM-TWH are not given in Figures 9*∼*11, and only the segmentation thresholds are summarized in the TWH column given in Table 2. The segmentation results of J_SB_MM-TDH with *n* = 6, 8, 11, and 13 are shown in Figures 9(a)∼9(d), respectively. Figures 9(e)∼9(n) show the segmentation thresholds of the left and right parts with *n* = 6∼15, respectively. Figures 10(a)∼10(n) and 11(a)∼11(n) give the corresponding segmentation results and thresholds of J_SB_MM-TDH for the middle and lower slices, respectively.

The segmentation thresholds with *n* = 6∼15 for the upper, middle, and lower slices are summarized in the corresponding TDH column given in Table 2. It is obvious that the segmentation thresholds almost tend to be stable when *n* is bigger than 12. While the segmentation thresholds in TWH column are also changeable, even *n* is bigger than 12, which is similar to the trend of GMM. By analyzing and comparing the range of segmentation thresholds between J_SB_MM-TDH and J_SB_MM-TWH with the same *n*, it can be seen that most of the upper limit values are close to each other, but the lower limit values of J_SB_MM-TDH are smaller than that of J_SB_MM-TWH, and the differences are mostly around 10.

Analyzing and comparing the segmentation results of (a)∼(d) shown in Figures 9∼11, respectively, the better segmentation results can be obtained for the upper, middle, and lower slices when *n* is 13. Therefore, considering the trend of segmentation thresholds given in Table 2, we determine to take *n* = 13 as the fixed cluster number for J_SB_MM-TDH to segment different CT image sequences in the following segmentation experiments in Section 4.

As a matter of convenience in comparison, Table 2 also gives the segmentation thresholds of GMM for liver CT sequence S1 shown in Table 1. By analyzing and comparing the range of segmentation thresholds between J_SB_MM-TWH and GMM with the same *n*, it is found that most of the upper and lower limit values are close to each other, which means the segmentation results of J_SB_MM-TWH are similar to that of GMM. Therefore, the segmentation results of J_SB_MM-TDH are both better than the results of J_SB_MM-TWH and GMM.

Table 3 gives the segmentation calculation time with different cluster numbers as shown in Figures 9–11. The segmentation time is less affected by the different cluster numbers, and it almost tends to decrease for the middle slice of Figure 10 with a large liver area. In this study, only the parameters Φ, *δ*, and *γ* are used to calculate the threshold value of analytic solution, so the segmentation speed is quite fast, and the effect of segmentation time with different cluster numbers can be ignored.

## 4. Segmentation Experimental Results

The J_SB_MM-TDH was applied to segment four randomly obtained abdominal CT image sequences from different image databases [47,48], and the segmentation thresholds and results of J_SB_MM-TDH are compared with that of GMM, as shown in Figures 12∼14, which are the upper, middle, and lower slices of the four different CT image sequences, respectively. In these figures, the first row shows the original image from four different CT image sequences, the second row gives the threshold segmentation results of GMM, and the third row is the binary images obtained according to the segmentation results of GMM. The fourth row shows the binary images obtained depending on the segmentation results of J_SB_MM-TDH. The fifth row is the segmentation results of GMM, and the sixth row gives the results of J_SB_MM-TDH. The seventh row and the last row provide the left and right segmentation thresholds of J_SB_MM-TDH, respectively.

Table 4 gives the comparison of segmentation thresholds and quantitative evaluation for Figures 12–14, respectively. Here, it needs to be stated that the segmentation results of GMM are fitted with different cluster numbers, which is the best one chosen from the segmentation results with *n* = 6∼15 for each slice for the sequences S2, S3, S4, and S5, respectively, while all segmentation results of J_SB_MM-TDH are fitted with the same cluster number *n* = 13. However, most segmentation results of J_SB_MM-TDH are better than those of GMM, and the other few results are similar to each other. On the whole, it is illustrated that not only the segmentation results of J_SB_MM-TDH are better than those of GMM, but also the cluster numbers can be fixed at *n* = 13 without worrying about overfitting. This is good for the implementation of automatic segmentation of liver CT images.

The Jaccard index and Dice coefficient are common indexes for quantitative evaluation of image segmentation. The Jaccard index is a statistic used for comparing the similarity of sample sets. The Dice coefficient is another similarity measure index. The Jaccard index and Dice coefficient are calculated to quantitatively evaluate the segmentation results of GMM and J_SB_MM-TDH, respectively. The values of the Jaccard index and Dice coefficient are given in Table 4, and the values in the column of difference mean the difference value between J_SB_MM-TDH and GMM, that is, the Jaccard index (or Dice coefficient) of J_SB_MM-TDH minus that of GMM. The last row gives the average value. The maximum value of difference column in the Jaccard index is 0.1987, and the average value of this column is 0.0691. The maximum value of difference column in the Dice coefficient is 0.1863, and the average value of this column is 0.048. By comprehensive quantitative comparison, it is found that the segmentation results of J_SB_MM-TDH are better than that of GMM.

The website addresses of the data sets S1, S2, S3, S4, and S5 are provided in Appendix B.

## 5. Conclusions

The J_SB_MM-TDH with flexibly skewed characteristics proposed in this study is suitable for fitting the skewness distribution of the gray-level histogram of liver CT images. The parameter optimization algorithm employing EM and the implementation process of the segmentation algorithm has been given in detail. The effects of cluster number on segmentation threshold were discussed and compared for GMM, J_SB_MM-TWH, and J_SB_MM-TDH, respectively. It is shown that the J_SB_MM-TDH threshold will tend to be stable at cluster number 13, while the threshold of GMM and the threshold of J_SB_MM-TWH are similar and sensitive to different cluster numbers. The proposed J_SB_MM-TDH with cluster number 13 is applied to segment four random CT image sequences, and the segmentation results are compared with those of GMM. Analyzing the segmentation results and quantitative evaluations, it is further illustrated that J_SB_MM-TDH does not have the overfitting phenomenon with the increase in cluster number, which verifies that J_SB_MM-TDH has preferable segmentation results and better robustness than GMM. J_SB_MM-TDH makes it possible to realize the automatic segmentation of live CT image due to the robustness with the fixed cluster number. The J_SB_MM-TDH can be used not only for liver CT image segmentation, but also for other CT image segmentation as well.

## Figures and Tables

**Figure 1:** Probability density of normal, gamma, exponential, Student's *t*, and Rayleigh distributions. (a) *μ* : mean, *σ* : standard deviation. (b) *α* : shape parameter, *β* : scale parameter. (c) *μ* : mean. (d) *x* : position parameter, *ν* : degrees of freedom. (e) *B*: scale parameter.

**Figure 2:** Upper, middle, and lower slices of the liver CT image and their histograms. (a) The upper slice. (b) The middle slice. (c) The lower slice. (d) Gray-level histogram of (a). (e) Gray-level histogram of (b). (f) Gray-level histogram of (c).

**Figure 3:** Probability density function curves with different parameters.

**Figure 4:** Frontal outline and the upper, middle, and lower sections of the liver CT scan sequence.

**Figure 5:** Slices of 1/3 of the liver and the corresponding LV_A. (a) A slice of 1/3 of the liver in the first sequence. (b) The LV_A of (a) is 131. (c) A slice of 1/3 of the liver in the second sequence. (d) The LV_A of (b) is 178.

**Figure 6:** Maximum gray value of the liver (LV_M) in CT slice image. (a) The upper section. (b) LV_M of Figure 6(a), (c) The lower section. (d) LV_M of Figure 6(c).

**Figure 7:** Grayscale values of segmentation points and the binarized result.

**Figure 8:** Segmentation results and thresholds of GMM with different cluster numbers. (a) *n* *=* 6. (b) *n* *=* 8. (c) *n* *=* 10. (d) *n* *=* 12. (e) *n* *=* 14.

**Figure 9:** Segmentation thresholds of JSBMM-TDH with different cluster numbers for the upper slice. (a) *n* = 6. (b) *n* = 8. (c) *n* = 11. (d) *n* = 13. (e) *n* = 6. (f) *n* = 7. (g) *n* = 8. (h) *n* = 9. (i) *n* = 10. (j) *n* = 11. (k) *n* = 12. (l) *n* = 13. (m) *n* = 14. (n) *n* = 15.

**Figure 10:** Segmentation thresholds of JSBMM-TDH with different cluster numbers for the middle slice. (a) *n* = 6. (b) *n* = 8. (c) *n* = 11. (d) *n* = 13. (e) *n* = 6. (f) *n* = 7. (g) *n* = 8. (h) *n* = 9. (i) *n* = 10. (j) *n* = 11. (k) *n* = 12. (l) *n* = 13. (m) *n* = 14. (n) *n* = 15.

**Figure 11:** Segmentation thresholds of JSBMM-TDH with different cluster numbers for the lower slice. (a) *n* = 6. (b) *n* = 8. (c) *n* = 11. (d) *n* = 13. (e) *n* = 6. (f) *n* = 7. (g) *n* = 8. (h) *n* = 9. (i) *n* = 10. (j) *n* = 11. (k) *n* = 12. (l) *n* = 13. (m) *n* = 14. (n) *n* = 15.

**Figure 12:** Binary images, segmentation thresholds, and results of J_SB_MM-TDH and GMM for the upper slice.

**Figure 13:** Binary images, segmentation thresholds, and results of J_SB_MM-TDH and GMM for the middle slice.

**Figure 14:** Binary images, segmentation thresholds, and results of J_SB_MM-TDH and GMM for the lower slice.

**Algorithm 1:** EM algorithm for JSBMM.

**Algorithm 2:** Segmentation algorithm based on J_SB_MM.

**Table 1:** Segmentation thresholds of two different CT image sequences using GMM.

Cluster number (*n*)	Segmentation thresholds					
	Slices of sequence S1			Slices of sequence S2		
	Upper	Middle	Lower	Upper	Middle	Lower
6	153∼201	168∼196	158∼204	115∼149	117∼149	115∼147
7	157∼201	168∼195	162∼194	109∼150	117∼150	115∼148
8	153∼202	165∼197	157∼196	122∼148	121∼145	120∼144
9	175∼193	169∼197	175∼188	112∼149	117∼152	116∼148
10	154∼201	172∼190	158∼196	124∼150	122∼150	121∼145
11	173∼195	169∼193	168∼191	113∼148	118∼153	116∼149
12	174∼194	168∼194	169∼191	126∼150	124∼150	124∼147
13	177∼193	172∼184	168∼189	115∼147	117∼150	116∼149
14	173∼194	169∼190	166∼191	127∼150	124∼150	125∼146
15	173∼194	168∼193	168∼191	117∼144	118∼142	117∼145

**Table 2:** Segmentation thresholds of S1 with different segmentation methods.

*n*	The upper slice			The middle slice			The lower slice		
	J_SB_MM		GMM (Figure 8)	J_SB_MM		GMM (Figure 8)	J_SB_MM		GMM (Figure 8)
	TDH (Figure 9)	TWH		TDH (Figure 10)	TWH		TDH (Figure 11)	TWH	
6	143∼194	157∼194	153∼201	166∼200	167∼195	168∼196	149∼189	160∼194	158∼204
7	147∼194	156∼198	157∼201	162∼199	171∼190	168∼195	148∼195	161∼193	162∼194
8	159∼194	164∼193	153∼202	162∼198	168∼195	165∼197	151∼195	165∼192	157∼196
9	160∼194	176∼192	175∼193	162∼196	168∼196	169∼197	153∼196	170∼190	175∼188
10	160∼194	176∼192	154∼201	161∼195	173∼190	172∼190	156∼196	171∼187	158∼196
11	161∼194	175∼192	173∼195	162∼194	170∼187	169∼193	156∼190	168∼189	168∼191
12	163∼193	175∼193	174∼194	162∼194	171∼188	168∼194	157∼189	170∼189	169∼191
13	**164∼194**	176∼193	177∼193	**161∼193**	171∼189	172∼184	**157∼188**	171∼189	168∼189
14	**164∼194**	177∼192	173∼194	**161∼193**	171∼185	169∼190	**158∼188**	169∼186	166∼191
15	**164∼194**	172∼185	173∼194	**162∼193**	171∼186	168∼193	**158∼188**	170∼188	168∼191

It is obvious that the segmentation thresholds almost tend to be stable when *n* is bigger than 12, which is shown as the bold values shown in TDH columns.

**Table 3:** Segmentation calculation time for the J_SB_MM with TDH for the upper, middle, and lower slices when *n* *=* 6∼15, respectively (time unit is second).

*n*	6	7	8	9	10	11	12	13	14	15
Upper (Figure 9)	2.62	11.7	5.71	3.05	3.30	5.60	3.01	4.89	5.15	1.99
Middle (Figure 10)	5.09	6.26	5.51	4.58	4.97	4.46	4.03	3.64	3.94	3.64
Lower (Figure 11)	2.41	7.57	4.38	2.59	3.09	2.95	2.56	4.10	5.41	3.47

**Table 4:** Comparison of segmentation thresholds and quantitative evaluation for Figures 12–14.

Liver slice position	Sequence	Segmentation thresholds		Quantitative evaluation					
		GMM	JSBMM-TDH(*n* = 13)	Jaccard index			Dice's coefficient		
				GMM	JSBMM-TDH	Difference	GMM	JSBMM-TDH	Difference
Upper slice (Figure 12)	S2	126∼150 (*n* = 12)	126∼146	0.9063	0.8854	−0.0209	0.9509	0.9392	−0.0117
	S3	152∼169 (*n* = 12)	146∼171	0.8793	0.9483	0.069	0.9358	0.9735	0.0377
	S4	127∼143 (*n* = 12)	122∼152	0.5955	0.7608	0.1653	0.7465	0.8641	0.1176
	S5	196∼226 (*n* = 12)	181∼212	0.5818	0.7805	0.1987	0.7356	0.8767	0.1411

Middle slice (Figure 13)	S2	123∼154 (*n* = 12)	117∼144	0.9173	0.9298	0.0125	0.9569	0.9636	0.0067
	S3	152∼173 (*n* = 13)	149∼177	0.9549	0.948	−0.0069	0.9769	0.9733	−0.0036
	S4	130∼145 (*n* = 12)	108∼151	0.6523	0.9527	0.3004	0.7895	0.9758	0.1863
	S5	188∼221 (*n* = 11)	172∼213	0.9744	0.9744	0.0	0.9501	0.9501	0.0

Lower slice (Figure 14)	S2	125∼151 (*n* = 12)	125∼140	0.8852	0.8794	−0.0058	0.9391	0.9358	−0.0033
	S3	158∼170 (*n* = 14)	149∼175	0.8234	0.904	0.0806	0.9031	0.9496	0.0465
	S4	100∼126 (*n* = 13)	113∼153	0.8715	0.8777	0.0062	0.9314	0.9349	0.0035
	S5	192∼223 (*n* = 11)	169∼212	0.9422	0.9719	0.0297	0.8907	0.9454	0.0547

Average value				0.832	0.9011	0.0691	0.8922	0.9402	0.048

## Data Availability

The DICOM data used to support the findings of this study have been deposited in the CHAOS repository (https://doi.org/10.5281/zenodo.3362844) and FAIRsharing repository (https://doi.org/10.25504/FAIRsharing.jrfd8y).

## Appendix

### A

M-step updates equations (6)*∼*(8) for solving the JSBMM parameters presented in Section 2.2.2, which are derived by maximizing the complete data log-likelihood *Q* with respect to each model parameter as follows:

(A.1) $$\begin{array}{c} \text{Q}\left(\theta_{k}\right)=\overset{N}{\underset{i=1}{\sum }}\overset{K}{\underset{k=1}{\sum }}{\text{P}}_{i,k}\left\{\text{ln}\Phi_{k}+{\text{ln}\delta }_{\text{k}}+\text{ln}\frac{\lambda }{\sqrt{2\pi }\left(x_{i}-\xi \right)\left(\lambda +\xi -x_{i}\right)}-\;\frac{1}{2}{\left[\gamma_{k}+\delta_{k}\text{ln}\left(\frac{x_{i}-\xi }{\lambda +\xi -x_{i}}\right)\right]}^{2}\right\}. \end{array}$$

(A.2) $$\begin{array}{c} \frac{\partial Q}{\partial \gamma_{k}}=\overset{N}{\underset{i=1}{\sum }}{\text{P}}_{i,k}\left[-\left(\gamma_{k}+\delta_{k}\text{ln}\left(\frac{x_{i}-\xi }{\lambda +\xi -x_{i}}\right)\right)\right]=-\left\{\gamma_{k}\overset{N}{\underset{i=1}{\sum }}{\text{P}}_{i,k}+\delta_{k}\overset{N}{\underset{i=1}{\sum }}\left[{\text{P}}_{i,k}\text{ln}\left(\frac{x_{i}-\xi }{\lambda +\xi -x_{i}}\right)\right]\right\}. \end{array}$$

Let

(A.3) $$\begin{array}{c} \frac{\partial Q}{\partial \gamma_{k}}=0. \end{array}$$

Then,

(A.4) $$\begin{array}{c} \gamma_{k}=-\frac{\sum_{i=1}^{N}\left[{\text{P}}_{i,k}\text{ln}\left(x_{i}-\xi /\lambda +\xi -x_{i}\right)\right]}{\sum_{i=1}^{N}{\text{P}}_{i,k}}\delta_{k}=-\frac{A}{B}\delta_{k}, \end{array}$$

where

(A.5) $$\begin{array}{c} \text{A}=\overset{N}{\underset{i=1}{\sum }}\left[{\text{P}}_{i,k}\text{ln}\left(\frac{x_{i}-\xi }{\lambda +\xi -x_{i}}\right)\right]\text{,}\;\text{B}=\overset{N}{\underset{i=1}{\sum }}{\text{P}}_{i,k}. \end{array}$$

(A.6) $$\begin{array}{c} \frac{\partial Q}{\partial \delta_{k}}=\overset{N}{\underset{i=1}{\sum }}{\text{P}}_{i,k}\left[\frac{1}{\delta_{k}}-\left(\gamma_{k}+\delta_{k}\text{ln}\left(\frac{x_{i}-\xi }{\lambda +\xi -x_{i}}\right)\right)\text{ln}\left(\frac{x_{i}-\xi }{\lambda +\xi -x_{i}}\right)\right]. \end{array}$$

(A.7) $$\begin{array}{c} ∵\gamma_{k}=-\frac{A}{B}\delta_{k}. \end{array}$$

(A.8) $$\begin{array}{c} ∴\;\frac{\partial Q}{\partial \delta_{k}}=\overset{N}{\underset{i=1}{\sum }}{\text{P}}_{i,k}\left[\frac{1}{\delta_{k}}-\left(-\frac{A}{B}\delta_{k}+\delta_{k}\text{ln}\left(\frac{x_{i}-\xi }{\lambda +\xi -x_{i}}\right)\right)\text{ln}\left(\frac{x_{i}-\xi }{\lambda +\xi -x_{i}}\right)\right]=\overset{N}{\underset{i=1}{\sum }}{\text{P}}_{i,k}\left[\frac{1-\left(-A/B+\text{ln}\left(x_{i}-\xi /\lambda +\xi -x_{i}\right)\right)\delta_{k}^{2}\text{ln}\left(x_{i}-\xi /\lambda +\xi -x_{i}\right)}{\delta_{k}}\right]. \end{array}$$

Let

(A.9) $$\begin{array}{c} \frac{\partial Q}{\partial \delta_{k}}=0. \end{array}$$

Then,

(A.10) $$\begin{array}{c} \overset{N}{\underset{i=1}{\sum }}{\text{P}}_{i,k}\left[1-\left(-\frac{A}{B}+\text{ln}\left(\frac{x_{i}-\xi }{\lambda +\xi -x_{i}}\right)\right)\delta_{k}^{2}\text{ln}\left(\frac{x_{i}-\xi }{\lambda +\xi -x_{i}}\right)\right]=0. \end{array}$$

(A.11) $$\begin{array}{c} \overset{N}{\underset{i=1}{\sum }}{\text{P}}_{i,k}\left[1-\left(-\frac{A}{B}+\text{ln}\left(\frac{x_{i}-\xi }{\lambda +\xi -x_{i}}\right)\right)\delta_{k}^{2}\text{ln}\left(\frac{x_{i}-\xi }{\lambda +\xi -x_{i}}\right)\right]=0\\ \Rightarrow \delta_{k}^{2}=\frac{\sum_{i=1}^{N}{\text{P}}_{i,k}}{\sum_{i=1}^{N}{\text{P}}_{i,k}\left[\left(-A/B+\text{ln}\left(x_{i}-\xi /\lambda +\xi -x_{i}\right)\right)\text{ln}\left(x_{i}-\xi /\lambda +\xi -x_{i}\right)\right]}\\ =\frac{\sum_{i=1}^{N}{\text{P}}_{i,k}}{-A/B\sum_{i=1}^{N}\left[{\text{P}}_{i,k}\text{ln}\left(x_{i}-\xi /\lambda +\xi -x_{i}\right)\right]+\sum_{i=1}^{N}\left[{\text{P}}_{i,k}{\text{ln}}^{2}\left(x_{i}-\xi /\lambda +\xi -x_{i}\right)\right]}=\frac{B}{\sum_{i=1}^{N}\left[{\text{P}}_{i,k}{\text{ln}}^{2}\left(x_{i}-\xi /\lambda +\xi -x_{i}\right)\right]-A^{2}/B}=\frac{B}{C-A^{2}/B}. \end{array}$$

where

(A.12) $$\begin{array}{c} \text{C}=\overset{N}{\underset{i=1}{\sum }}\left[{\text{P}}_{i,k}{\text{ln}}^{2}\left(\frac{x_{i}-\xi }{\lambda +\xi -x_{i}}\right)\right],\;\delta_{k}^{2}=\frac{B}{C-A^{2}/B}=\frac{B^{2}}{BC-A^{2}}. \end{array}$$

*BC* − *A*^2^ > 0 is proved, because

(A.13) $$\begin{array}{c} \text{A}=\overset{N}{\underset{i=1}{\sum }}\left[{\text{P}}_{i,k}\text{ln}\left(\frac{x_{i}-\xi }{\lambda +\xi -x_{i}}\right)\right]\;\text{B}=\overset{N}{\underset{i=1}{\sum }}{\text{P}}_{i,k}\;\text{C}=\overset{N}{\underset{i=1}{\sum }}\left[{\text{P}}_{i,k}{\text{ln}}^{2}\left(\frac{x_{i}-\xi }{\lambda +\xi -x_{i}}\right)\right]. \end{array}$$

Let

(A.14) $$\begin{array}{c} \text{ln}\left(\frac{x_{i}-\xi }{\lambda +\xi -x_{i}}\right)=X_{i}. \end{array}$$

Then,

(A.15) $$\begin{array}{c} BC-A^{2}=\left[\overset{N}{\underset{i=1}{\sum }}{\text{P}}_{i,k}\;\overset{N}{\underset{i=1}{\sum }}\left({\text{P}}_{i,k}X_{i}^{2}\right)\right]-{\left[\overset{N}{\underset{i=1}{\sum }}\left({\text{P}}_{i,k}{\text{X}}_{i}\right)\right]}^{2}\\ =\overset{N-1}{\underset{i=1}{\sum }}\overset{N}{\underset{j=i+1}{\sum }}P_{i,k}P_{j,k}{\left({\text{X}}_{i}-{\text{X}}_{j}\right)}^{2}. \end{array}$$

(A.16) $$\begin{array}{c} ∴BC-A^{2}>0. \end{array}$$

We have

(A.17) $$\begin{array}{c} \overset{K}{\underset{k=1}{\sum }}\Phi_{k}=1. \end{array}$$

Φ_*k*_ is solved by applying the method of Lagrange multipliers as follows:

(A.18) $$\begin{array}{c} \frac{\partial Q}{\partial \Phi_{k}}=\overset{N}{\underset{i=1}{\sum }}{\text{P}}_{i,k}\frac{1}{\Phi_{k}}+\alpha \\ \frac{\partial Q}{\partial \Phi_{k}}=0\;\Rightarrow \overset{N}{\underset{i=1}{\sum }}{\text{P}}_{i,k}\frac{1}{\Phi_{k}}=-\alpha \Rightarrow \overset{N}{\underset{i=1}{\sum }}{\text{P}}_{i,k}\frac{1}{\alpha }=-\Phi_{k}\Rightarrow \overset{K}{\underset{k=1}{\sum }}\overset{N}{\underset{i=1}{\sum }}{\text{P}}_{i,k}\frac{1}{\alpha }=-\overset{K}{\underset{k=1}{\sum }}\Phi_{k}\Rightarrow \overset{K}{\underset{k=1}{\sum }}\overset{N}{\underset{i=1}{\sum }}{\text{P}}_{i,k}\frac{1}{\alpha }=-1\Rightarrow \alpha =-\frac{1}{N}\\ \;\Phi_{k}=\frac{\sum_{i=1}^{N}{\text{P}}_{i,k}}{N}=\frac{B}{N}. \end{array}$$

### B

The data sets S1, S2, S3, S4, and S5 are from the following website address, respectively:

1. Data sets S2 and S4 are from the following website:
2. https://wiki.cancerimagingarchive.net/download/attachments/6885436/doiJNLP-TCGA-LIHC-01-30-2017.tcia?version=1&modificationDate=1534786974574&api=v2.
3. Data sets S1, S3, and S5 are from the following website:
4. https://zenodo.org/record/3431873/files/CHAOS_Train_Sets.zip?download=1.
